The article "Massively parallel sequencing and genome-wide copy number analysis revealed a clonal relationship in benign metastasizing leiomyoma" was published in 2017. Journal: Oncotarget.

# Massively parallel sequencing and genome-wide copy number analysis revealed a clonal relationship in benign metastasizing leiomyoma

**DOI:** 10.18632/oncotarget.17708

**Published:** 2017-05-09

**Authors:** Ren-Chin Wu, An-Shine Chao, Li-Yu Lee, Gigin Lin, Shu-Jen Chen, Yen-Jung Lu, Huei-Jean Huang, Chi-Feng Yen, Chien Min Han, Yun-Shien Lee, Tzu-Hao Wang, Angel Chao

**Affiliations:** ^1^ Department of Pathology, Chang Gung Memorial Hospital and Chang Gung University, Linkou Medical Center, Taoyuan, Taiwan; ^2^ Department of Obstetrics and Gynecology, Chang Gung Memorial Hospital and Chang Gung University, Linkou Medical Center, Taoyuan, Taiwan; ^3^ Department of Medical Imaging and Intervention, Clinical Phenome Center, Chang Gung Memorial Hospital and Institute for Radiological Research, Chang Gung University, Linkou Medical Center, Taoyuan, Taiwan; ^4^ ACT Genomics, Co. Ltd., Taipei City, Taiwan; ^5^ Gynecologic Cancer Research Center, Chang Gung Memorial Hospital, Taoyuan, Taiwan; ^6^ Department of Biotechnology, Ming-Chuan University, Taoyuan, Taiwan

**Keywords:** benign metastasizing leiomyoma, massively parallel sequencing, clonality, molecular inversion probe array

## Abstract

Benign metastasizing leiomyoma (BML) is a rare disease entity typically presenting as multiple extrauterine leiomyomas associated with a uterine leiomyoma. It has been hypothesized that the extrauterine leiomyomata represent distant metastasis of the uterine leiomyoma. To date, the only molecular evidence supporting this hypothesis was derived from clonality analyses based on X-chromosome inactivation assays. Here, we sought to address this issue by examining paired specimens of synchronous pulmonary and uterine leiomyomata from three patients using targeted massively parallel sequencing and molecular inversion probe array analysis for detecting somatic mutations and copy number aberrations. We detected identical non-hot-spot somatic mutations and similar patterns of copy number aberrations (CNAs) in paired pulmonary and uterine leiomyomata from two patients, indicating the clonal relationship between pulmonary and uterine leiomyomata. In addition to loss of chromosome 22q found in the literature, we identified additional recurrent CNAs including losses of chromosome 3q and 11q. In conclusion, our findings of the clonal relationship between synchronous pulmonary and uterine leiomyomas support the hypothesis that BML represents a condition wherein a uterine leiomyoma disseminates to distant extrauterine locations.

## INTRODUCTION

Benign metastasizing leiomyoma (BML), a rare disease entity of women, typically presents as extrauterine leiomyomas associated with a previously or synchronously diagnosed uterine leiomyoma [1]. The lungs are the predominant site of involvement, although other extrauterine sites including heart [2], bone [3], soft tissue, and lymph nodes have also been reported [4].

The origin of BML has been controversial. As implied by its name, BML has been hypothesized to be peculiar manifestation of a subgroup of uterine leiomyomas, which are capable of distant metastasis through hematogenous spread. Whereas metastasis is one of the defining traits of malignant neoplasm, BML generally has an indolent clinical course and histopathological features typical of a benign smooth muscle neoplasm. This incongruity has led to alternative hypothesis of the origin of BML, with some studies suggesting that BML represents a borderline tumor or a tumor with low malignant potential [5] whereas others have proposed that BML constitutes a manifestation of primary pulmonary leiomyomatosis clonally unrelated to the co-existing uterine leiomyoma [6].

To settle this issue, X-chromosome inactivation analysis has been employed to investigate the clonal relationship between the uterine and extrauterine leiomyomata [5, 7, 8]. These studies demonstrated identical X-chromosome inactivation pattern between uterine and extrauterine leiomyomata in four patients with BML, suggesting a clonal relationship. It should be noted, however, that a 50% chance exists of two random tumors exhibiting concordant X-chromosome inactivation pattern [5]. Therefore, the probability of observing 4 tumor pairs that showed concordant X-inactivation is theoretically 1/2^4^ (*p* = 0.0625), which is not sufficient to confidently refute the null hypothesis that the uterine and extrauterine tumors are not related clonally.

In the current study, we compared the clinicopathological features of three pairs of synchronous pulmonary and uterine and leiomyomata and applied targeted massively parallel sequencing and molecular inversion probe array analysis, with the aim of demonstrating the clonal relationship and discovering relevant genetic aberrations in BML.

## RESULTS

### Clinicopathological characteristics of three patients with BML

Three patients diagnosed with BML all presented with multiple pulmonary nodules characterized by bland-looking spindle tumor cells showing smooth muscle differentiation. Uterine leiomyomata were found in all patients shortly after the identification of pulmonary nodules. The clinical, histopathological, and immunohistochemical features of the cases are summarized in Table 1 and detailed as follows.

**Table 1:** Clinicopathological and immunohistochemical analyses of three pairs of synchronous uterine and lung leiomyomas

	case 1	case 2	case 3
Age (years)	35	37	46
Interval (months)^a^	−2 (lung first)	−1(lung first)	0 (simultaneously)
Largest lung tumor (mm)	13	9	36
Number of lung tumors	miliary	multiple	multiple
Atypia	Negative	Negative	Negative
Necrosis	Negative	Negative	Negative
Mitosis	Negative	Negative	Negative
ER	Positive	Positive	Positive
PR	Positive	Positive	Positive
SMA	Positive	Positive	Positive
desmin	Positive	Positive	Positive
CD34	Negative	Negative	NA
CD10	Negative	NA	focal
S-100	Negative	Negative	NA
HMB-45	Negative	NA	NA
CD117	NA	Negative	Negative

^a^ Interval between the detection of lung tumors and uterine tumor

NA: not applicable.

Case 1, a 35-year-old female without any symptoms, was found to have pulmonary lesions by chest X-ray in a routine health examination. A computed tomography (CT) scan revealed multiple well-defined, contrast-enhanced nodules in the peripheral parts of both lungs (Figure 1). She underwent thoracoscopic wedge resection of the largest pulmonary nodule, which measured 13 mm in the greatest dimension. The nodules were composed of fascicles of bland-looking spindle tumor cells without necrosis or mitotic figures. Immunohistochemically, the tumor cells showed cytoplasmic staining for smooth muscle actin (SMA) and desmin, and nuclear staining for estrogen receptor (ER) and progesterone receptor (PR). Following referral for gynecologic assessment, she was identified as having two uterine myometrial tumors and underwent laparoscopic myomectomy 2 months after detection of the lung nodules. The resected myometrial tumors, measuring 7 cm and 2 cm in the greatest dimension, exhibited similar histology to the pulmonary nodules and were characterized by fascicles of bland-appearing spindle cells with smooth muscle differentiation. She had been closely followed up for seven years with no progression of the number and/or size of the lung nodules having been noted.

**Figure 1:** Representative case of a synchronous lung and uterine leiomyomata (case 1) (**A**) Computed tomography scan displaying multiple, well-defined nodules in randomized distribution over bilateral lung bases. The maximal dimension of the nodules is 13 mm (red arrows). (**B**) Photomicrograph of a pulmonary leiomyoma. The inset shows that the pulmonary leiomyoma was composed of fascicles of bland-looking spindle cells. (**C**) Synchronous uterine leiomyoma exhibiting similar histology as the pulmonary leiomyoma. Immunohistochemically, the pulmonary leiomyoma was diffusely positive for (**D**) estrogen receptor and (**E**) progesterone receptor.

Case 2 was a 37-year-old female suffering from exertional dyspnea and a bearing-down sensation. Laboratory examination showed mild anemia (hemoglobin 11.6 g/dL). A CT scan revealed bilateral multiple lung nodules measuring 9 mm in the greatest dimension. The largest nodules over the upper and lower lung lobes were excised by thoracoscopic wedge resection. These nodules were composed of fascicles of spindle tumor cells without nuclear atypia or necrosis. The tumor cells showed positive immunostaining for SMA, desmin, ER, and PR. One month later, the patient received laparoscopy-assisted vaginal hysterectomy, which yielded a uterine leiomyoma measuring 7 cm in the maximum dimension. During three years of follow-up, there had been no newly developed lung nodules, although the remaining lung nodules increased in size slightly. The patient remained symptom free since the surgeries.

Case 3 was a 46-year-old female presenting with chronic productive cough and dyspnea. She also suffered from intermittent hypermenorrhea and severe anemia (hemoglobin 5.4 g/dL). A CT scan showed multiple pulmonary nodules with the largest (3.6 cm in dimension) being located in the left lingual lobe. Pathological examination of a CT-guided biopsy revealed tumor fragments consisting of bland-looking spindle cells immunoreactive to SMA, desmin, ER, and PR. Concomitantly, the patient underwent total abdominal hysterectomy for an enlarged uterus of 14 cm. Histopathological examination revealed adenomyosis and six leiomyomatous nodules. She received Leuplin Depot for six courses (3.75 mg intramuscular injection every month) to relieve her dyspnea. The pulmonary nodules remained stationary at six months after the operation. Her dyspnea improved by the two-year follow-up.

### Mutational analysis of synchronous pulmonary and uterine leiomyomata

Massively parallel sequencing for a panel of 409 cancer-related genes in this study identified 10 somatic mutations in the three pairs of synchronous pulmonary and uterine leiomyomata (Table 2). Evidence of a clonal relationship between pulmonary and uterine leiomyomata was observed in two patients (case 1 and 2). In case 1, the pulmonary and uterine leiomyomata shared three identical somatic mutations in *BCL11B* (c.1093C>T), *FANCD2* (c.1401_1402invGT), and *SYNE1* (c.19055C>T); whereas those of case 2 shared two somatic mutations in *DNMT3A* (c.2206C>T) and *MSH6* (c.1968C>G). In contrast, no shared somatic mutations were identified in case 3. No recurrently mutated genes were identified in this cohort of three BMLs. None of the aforementioned genes have been reported mutated in uterine leiomyoma.

**Table 2:** Single nucleotide variants and short insertion /deletions of three pairs of synchronous uterine and lung leiomyomas identified using a comprehensive cancer panel containing 409 cancer-related exons

Gene	DNA change	Protein change	case 1		case 2		case 3	
			Uterus	Lung	Uterus	Lung	Uterus	Lung
ATM	c.6198+3A>G	splice_region			0.0%	16.5%		
BCL11B	c.1093C>T	p.R365W	10.3%	5.2%				
DNMT3A	c.2206C>T	p.R736C			42.8%	28.8%		
FANCD2	c.1401_1402invGT	p.Y468H	7.5%	3.9%				
HCAR1	c.675G>T	p.V225V					0.0%	11.9%
LRP1B	c.3099C>A	p.D1033E	18.9%	0.0%				
MSH6	c.1968C>G	p.P656P			42.9%	25.4%		
MYH11	c.1402-2A>T	splice_acceptor					13.5%	0.0%
NTRK3	c.685A>G	p.I229V					0.0%	7.4%
SYNE1	c.19055C>T	p.A6423V	7.4%	3.4%				

Percentage indicates variant frequency of the mutation

### Genome-wide copy number analysis of synchronous pulmonary and uterine leiomyomata

The molecular inversion probe arrays also revealed similar patterns of copy number variations in the first two pairs of synchronous pulmonary and uterine leiomyomata, further suggestive of a clonal relationship (Figure 2). In case 1, both pulmonary and uterine leiomyomata were chromosomally stable without identified copy number aberrations (CNAs). Although this result was uninformative, it was consistent with the mutational analysis finding that the synchronous tumors in case 1 were clonally related. In case 2, three long-segment chromosomal losses involving chromosomes 3q13.31–3q29, 11q14.1–11q24.1, and 15q14–15q15.2 were identified in both pulmonary and uterine leiomyomata. The breakpoints of these segments in both tumors were identical or very close, highly suggestive of a clonal relationship (Figure 3). In case 3, the uterine tumor was chromosomally stable whereas the pulmonary tumor harbored a gain at chromosome 12q and losses at 6q and 14q. Thus, the clonality in this case remained undetermined.

**Figure 2:** Copy number variations in three pairs of synchronous pulmonary and uterine leiomyomata Blue and red blocks represent chromosome gains and losses, respectively. The synchronous tumors from case 2 shared three identical long-segment chromosome losses localized at chromosomes 3q, 11q, and 15q.

**Figure 3:** Details of the shared copy number variations identified in the uterine (left panel) and pulmonary (right panel) leiomyoma from case 2 For each aberrant chromosome, the chromosome ideograms (top), log2 ratio (middle), and B allele frequency (bottom) are shown. All three segments of chromosome loss (red bar) had identical or very close breakpoints between uterine and pulmonary leiomyomas.

## DISCUSSION

Although BML was first reported in 1939 [9], the rarity of this disease has limited our understanding of its origin and pathogenesis. The mainstream hypothesis is that BML represents a peculiar condition where a benign uterine leiomyoma spreads to distant extrauterine locations [1, 5, 10]. Our study applied massively parallel sequencing of a large panel of cancer-related genes, which revealed shared somatic mutations in two pairs of synchronous uterine and pulmonary leiomyomata (cases 1 and 2). Because none of the shared mutations were hot-spot mutations or genetic changes frequently found in leiomyoma, the probability of finding these genetic aberrations in two clonally unrelated tumors was extremely low. Our results provided concrete evidence of a clonal relationship between synchronous pulmonary and uterine leiomyomata, supporting the notion that BML represents extrauterine dissemination of uterine leiomyomas.

Consistent with the findings of targeted massively parallel sequencing, genome-wide copy number analysis revealed similar patterns of CNAs between pulmonary and uterine leiomyomata in cases 1 and 2. However, the clonality status of case 3 remained unknown as no shared single nucleotide variant, insertion/deletion, or CNAs were identified. It is possible that the synchronous tumors in case 3 were clonally related but that the shared clonal mutations were not identified owing to the limited breadth of sequencing coverage, which encompassed only the exons of 409 cancer-related genes. Whole exome or genome sequencing is likely required to determine the clonal relationship of the synchronous leiomyomata in case 3.

Our study was the first that applied massively parallel sequencing on BML samples. Although somatic mutations were identified in all cases, no recurrent mutations were observed in our small cohort of BML. Similarly, we did not identify recurrent CNAs by molecular inversion probe array. To identify recurrent CNAs in BML, we reviewed the English literature and found eight BMLs that have been investigated for CNA (Table 3) [7, 8, 10, 11]. Of the 11 BMLs studied (including three in the present study), chromosomal loss of 3q were found in three cases (27%) loss of 11q in two cases (18%), and loss of 22q in two cases (18%) (Table 3) [10, 11]. The overlapping genomic regions in these recurrent events, however, were too broad to identify candidate genes. To identify the aberrant, disease-causing pathways in BML, a much larger collection of samples examined with higher resolution platforms for copy number variations is required.

**Table 3:** Copy number aberrations (CNAs) of benign metastasizing leiomyomas in the literature and the present study

Author	Method	Number of cases	CNV^a^
Lin [8]	Single Nucleotide Polymorphism 6.0	1	No imbalance (2)
Bowen [11]	250K Nsp Assay Kits	1	Loss in 1p36.33–p36.23 (2),1p36.13–p35.2 (2), 2q37.3 (2), **3q23** (2), **3q25.1** (2), **3q25.32**–**q26.33** (2), 7p22.3–q31.33 (2), 10q22.3–q23.33 (2), and **22q11.1–q13.33 (2)**
Nucci [10]	Karyotyping	5	Gain in 1p11 (1), 1p21 (1), 1p35 (1), 2p25 (1), 6p21-p22 (1), 7q36 (1), 12q22-q24 (1), 13p10 (1), chr16 (1), 19q13 (1), 19q13.3 (1), 22q12 (1), 22q13 (1), chr22 (1) Loss in chr2 (1), **3q22** (1), 4p12 (1), 6p21 (1), chr8 (1), chr10 (1), **11q21-q23** (1), chr12, chr13 (2), chr14 (2), **chr22** (1)
Tietze [7]	Competitive hybridization of fluorescein isothiocyanate-labeled tumor DNA	1	No imbalance (2)
Present study	Molecular inversion probe array (OncoScan)	3	Loss in **3q13.31–q29** (2), **11q14.1–q24.1** (2), 15q14–q15.2 (2)

^a^ Brackets show the number of specimens.

Recurrent copy number aberrations are shown in block letters, i.e. chromosome 3q, 11q, and 22q.

Pulmonary BML lesions generally are indolent and asymptomatic as in two of the three patients in our series. Pulmonary BML usually exhibits a miliary pattern on radiologic scans that prompts surveying for interstitial or infectious diseases [1, 5, 10, 12]. Diagnosis of pulmonary BML is based on lung biopsies and/or resection of lung tumors. However, if symptoms appear in some cases such as hemoptysis, hemothorax, or a pneumothorax after diagnosis of BML, patients might benefit from hormonal treatment with luteinizing hormone-releasing hormone agonists such as leuprolide, aromatase inhibitors such as anastrozole, or raloxifene, a selective estrogen receptor modulator [13]. Similar hormonal manipulation was performed in case 3 of our study, as she suffered from exertional dyspnea that was ameliorated after treatment with leuprolide.

In summary, our genomic evidence deriving from massively parallel sequencing supported the clonal relationship between synchronous pulmonary and uterine leiomyomata. Thus, BML can be regarded as extrauterine spreading of uterine leiomyoma. However, the underlying mechanism that renders uterine leiomyomata capable of distant metastasis remains enigmatic. A more thorough genomic analysis on a much larger collection of BML samples is warranted to address this critical question.

## MATERIALS AND METHODS

### Patients

This study was approved by the IRB of Chang Gung Memorial Hospital (IRB Number: 103-4707B). Formalin-fixed paraffin-embedded (FFPE) specimens from three pairs of uterine and pulmonary leiomyomata were included. The corresponding buccal swabs of cases 1 and 3 as well as non-tumor FFPE specimens of case 2 were obtained.

### DNA isolation

DNA was extracted according to the protocols for isolation of total DNA from FFPE tissues and buccal swabs (Qiagen Inc., Valencia, CA, USA), as reported in our prior studies [14, 15]. Briefly, the cell pellet was obtained by centrifuging for 5 min at 300 × *g*. Samples were lysed by adding 20 μL proteinase K and 0.2 mL buffer AL and incubated at 56°C for 10 min. Then, 0.2 mL of 96–100% ethanol was added for precipitation. The sample mixture was loaded onto the DNeasy Mini Spin Column. After two wash steps, DNA solution was eluted and the aliquot was used for further analysis.

### Targeted massively parallel sequencing and data analysis

Sequencing procedures and data analysis were similar to those used in our previous reports [14, 15]. For each sample, 80 ng of genomic DNA was amplified by polymerase chain reaction using AmpliSeq Comprehensive Cancer Panel primer pools (Thermo Fisher Scientific, Waltham, MA, USA) to enrich the coding exons of 409 cancer-related genes. Amplicons were ligated with barcoded adaptors, conjugated with sequencing beads, and enriched using Ion Chef (Thermo Fisher Scientific) according to the Ion Torrent protocol. Sequencing was performed on the Ion Proton sequencer using the Ion PI chip (Thermo Fisher Scientific) according to the manufacturer's protocol. Raw data generated by the sequencer were mapped to the hg19 reference genome using Ion Torrent Suite (v. 4.2). Single nucleotide variants and short insertion/deletions were identified using the Torrent Variant Caller plug-in (v. 4.2). All variants were annotated using Variant Effect Predictor (VEP, release 78). Variants with less than 50 reads or variant frequency lower than 5% were filtered out. Variants were further annotated for COSMIC (v. 70), dbSNP (138), and 1000 Genomes (phase 1).

### Genome-wide copy number analysis by molecular inversion probe arrays

Molecular inversion probe arrays (OncoScan FFPE assay, Affymetrix, Santa Clara, CA, USA) were performed at the Genomic Medicine Research Core Laboratory, Chang Gung Memorial Hospital according to the manufacturer's protocol. The CNAs were analyzed using OncoScan Console 1.3 software and Nexus Express software for OncoScan 3.1. The SNP-FASST2 algorithm was used for segmentation and calling of chromosomal gains and losses with the following parameters: significance threshold = 5.0E^−11^, max contiguous probe spacing = 1000 Kbp, min number of probes per segment = 20, gain = 0.2, loss = −0.2. Chromosomal gains or losses smaller than 1.5 Mb were filtered.
